# Impact of overweight on left ventricular function in type 2 diabetes mellitus

**DOI:** 10.1186/s12933-017-0632-5

**Published:** 2017-11-09

**Authors:** Makiko Suto, Hidekazu Tanaka, Yasuhide Mochizuki, Jun Mukai, Hiroki Takada, Fumitaka Soga, Kumiko Dokuni, Yutaka Hatani, Keiko Hatazawa, Hiroki Matsuzoe, Hiroyuki Sano, Hiroyuki Shimoura, Junichi Ooka, Kensuke Matsumoto, Yushi Hirota, Wataru Ogawa, Ken-ichi Hirata

**Affiliations:** 1 Division of Cardiovascular Medicine, Department of Internal Medicine, Kobe University Graduate School of Medicine, 7-5-2, Kusunoki-cho, Chuo-ku, Kobe, 650-0017 Japan; 2 Division of Diabetes and Endocrinology, Department of Internal Medicine, Kobe University Graduate School of Medicine, Kobe, Japan

**Keywords:** Diabetes mellitus, Left ventricular longitudinal function, Left ventricular diastolic function, Obesity

## Abstract

**Background:**

Coexistence of left ventricular (LV) longitudinal myocardial systolic dysfunction with LV diastolic dysfunction could lead to heart failure with preserved ejection fraction (HFpEF). Diabetes mellitus (DM) is known as a significant factor associated with HFpEF. Although the mechanisms of DM-related LV myocardial injury are complex, it has been postulated that overweight contributes to the development of LV myocardial injury in type 2 diabetes mellitus (T2DM) patients. However, the precise impact of overweight on LV longitudinal myocardial systolic function in T2DM patients remains unclear.

**Methods:**

We studied 145 asymptomatic T2DM patients with preserved LV ejection fraction (LVEF) without coronary artery disease. LV longitudinal myocardial systolic function was assessed by global longitudinal strain (GLS), which was defined as the average peak strain of 18-segments obtained from standard apical views. Overweight was defined as body mass index (BMI) ≥ 25 kg/m^2^. Ninety age-, gender- and LVEF-matched healthy volunteers served as controls.

**Results:**

GLS of overweight T2DM patients was significantly lower than that of non-overweight patients (17.9 ± 2.4% vs. 18.9 ± 2.6%, p < 0.05), whereas GLS of both overweight and non-overweight controls was similar (19.8 ± 1.3% vs. 20.4 ± 2.1%, p = 0.38). Furthermore, multiple regression analysis revealed that for T2DM patients, BMI was the independent determinant parameters for GLS as well as LV mass index.

**Conclusions:**

Overweight has a greater effect on LV longitudinal myocardial systolic function in T2DM patients than on that in non-DM healthy subjects. Our finding further suggests that the strict control of overweight in T2DM patients may be associated with prevention of the development of HFpEF.

## Introduction

Heart failure (HF) with preserved ejection fraction (HFpEF), which is determined as the presence of HF symptoms and signs with left ventricular ejection fraction (LVEF) ≥ 50% [1], currently accounts for roughly half of all HF cases and its prevalence is related to HF with reduced ejection fraction (HFrEF). Patients with HFpEF usually are of advanced age and predominantly women with multiple comorbidities [2, 3], and diabetes mellitus (DM) is considered a major cause of HFpEF, accounting for 20–45% of all cases [4]. DM-related cardiac dysfunction is currently defined as a form of LV diastolic dysfunction, and several studies of DM patients have identified LV diastolic dysfunction as the earliest functional alteration in the course of diabetic cardiomyopathy [5–8], which could lead to the development of HFpEF. On the other hand, LV longitudinal myocardial systolic dysfunction has been identified in DM patients with preserved LVEF but without overt coronary artery disease or HF [9–16], and some investigators reported that it may be considered the first marker of a preclinical form of DM-related cardiac dysfunction in such patients [9, 17]. Thus, LV longitudinal myocardial systolic dysfunction may coexist with LV diastolic dysfunction in patients with DM and lead to HFpEF. It has been demonstrated that overweight is also an important cause of HFpEF as well as DM, with more than 80% of patients with HFpEF being overweight [18]. In addition, it has been postulated that overweight contributes to the development of LV myocardial injury in DM patients, but the precise impact of overweight on LV function is not yet fully understood. The aim of this study was thus to investigate the effect of overweight on LV longitudinal myocardial systolic function in asymptomatic patients with type 2 DM (T2DM) with preserved LVEF but without coronary artery disease.

## Methods

### Study population

Between July 2013 and September 2015, 155 asymptomatic T2DM patients admitted to Kobe University Hospital were prospectively enrolled in this study. Patients were excluded from enrolment study if they met any of the following criteria: (1) previous or current history of HF; (2) previous history or suspicion of coronary artery disease; (3) LVEF < 55%; (4) previous history of open-heart surgery and congenital heart disease; (5) serious renal dysfunction defined as glomerular filtration rate < 30 mL/min/1.73 m^2^; (6) uncontrolled hypertension > 180/100 mmHg; (7) more than moderate valvular heart disease; and (8) atrial fibrillation. All patients underwent exercise stress or pharmacological testing such as treadmill exercise or stress myocardial perfusion scintigraphy > 2 weeks after admission, and none of them showed an ischemic response. The diagnosis of T2DM was based on the World Health Organization criteria [19]. For comparison, a control group randomly taken from our database by the observers who have no involvement in echocardiographic analysis to have a similar age, gender and LVEF distribution, and consisting of 90 subjects without a history of DM or other cardiovascular disease. This study was approved by the local ethics committee of our institution (No. 160205).

### Echocardiographic examination

All patients underwent a resting standard echocardiographic examination less than 2 weeks after admission by means of a 3.5 MHz transducer on a single commercially available echocardiographic system (Vivid E9; General Electric Medical Systems, Milwaukee, WI). Digital routine grayscale two-dimensional cine loops from three consecutive heart beats were obtained at end-expiratory apnea from standard parasternal and apical views used for speckle-tracking strain analysis. Sector width was optimized to allow complete myocardial visualization while maximizing the frame rate. Standard echocardiographic measurements were obtained according to the current guidelines of the American society of echocardiography/European association of cardiovascular imaging [20]. Conventional LV diastolic function was also evaluated based on current guidelines [21].

### LV speckle-tracking strain analysis

Two-dimensional speckle-tracking strain analysis was semi-automatically performed with dedicated software (EchoPAC version 113; General Electric Medical Systems). Briefly, the first region of interest was manually traced with the point-and-click approach on the endocardium of LV at the end-systole phase. The second larger region of interest was then generated outside and carefully adjusted near the epicardium. Finally, six strain segments and corresponding time–strain curves were generated. We used the onset point of the QRS complex as a reference for LV strain analysis. Global longitudinal strain (GLS) was then determined as the averaged peak strain from three standard apical views in accordance with current guidelines (Fig. 1) [20], which also recommend expressing all strain values as absolute values, as was done in our study, to avoid confusion about magnitude relationships.

**Fig. 1:** Example of a color-coded two-dimensional display of the left ventricle (LV) and corresponding time–strain curves from 18 LV sites derived from the three standard apical views for measurement of global longitudinal strain (GLS). GLS was determined as the average peak strain of 18 LV segments, and was expressed as an absolute value

### Clinical data for T2DM patients

Dyslipidemia was defined as fasting low-density lipoprotein ≥ 140 mg/dL, or current use of anti-dyslipidemia drugs [22]. Blood pressure was obtained simultaneously with transthoracic echocardiography. Hypertension was then defined as systolic blood pressure ≥ 140 mmHg or diastolic blood pressure ≥ 90 mmHg, or current treatment with anti-hypertensive agents [23]. Overweight was defined in accordance with the World Health Organization’s definition as body mass index (BMI) ≥ 25 kg/m^2^.

### Statistical analysis

Continuous variables were expressed as mean values ± SD, while categorical data were summarized as frequencies and percentages. The parameters of the two subgroups were compared by using the unpaired t test, which was also used for comparison of continuous variables. Proportional differences were evaluated with the Chi square test and Fisher’s exact test. Independent associations of GLS with clinical and echocardiographic parameters in T2DM patients were evaluated by means of multiple regression analysis. The confounding factors for multiple regression analysis were based on the associated factors with subclinical LV dysfunctions in DM patients with preserved LVEF which were previously reported [14, 15, 24]. Statistical significance for each step was basically defined as p value < 0.05. All the analyses were performed with commercially available software (MedCalc software version 15.11.4; MedCalc Software, Mariakerke, Belgium).

## Results

### Baseline characteristics of T2DM patients and controls

Of the total of 155 T2DM patients enrolled in this study, 10 patients (6%) were excluded from all subsequent analyses because of suboptimal quality of echocardiographic images, so that the final study population consisted of 145 T2DM patients. The baseline characteristics of the latter and the 90 controls are summarized in Table 1. Clinical data showed that patients with T2DM were more likely to have higher BMI and heart rate, while echocardiographic data showed they were more likely to have a smaller stroke volume and GLS, and a larger left atrial volume index, LV mass index and E/e′. Table 2 shows the baseline characteristics of the T2DM patients with and without overweight. Overweight, defined as BMI ≥ 25 kg/m^2^, was detected in 75 T2DM patients (52%), and the remaining 70 (48%) were classified as T2DM patients without overweight. Clinical data showed that the prevalence of dyslipidemia in T2DM patients with overweight was higher than in those without overweight, while echocardiographic data showed that T2DM patients with overweight had a higher LV mass index and lower GLS compared to those without overweight. Intra- and inter-observer reproducibility for GLS for DM patients in our study group was previously reported [14–16, 24].

**Table 1:** Baseline characteristics of normal controls and T2DM patients

	Controls (n = 90)	T2DM patients (n = 145)	p value
Clinical data			
Age, years	57 ± 15	60 ± 13	0.08
Female, n (%)	50 (56)	67 (46)	0.16
Body mass index, kg/m^2^	22.0 ± 3.9	25.4 ± 5.0	< 0.05
Body mass index ≥ 25 kg/m^2^, n (%)	14 (16)	70 (48)	< 0.05
Body mass index ≥ 30 kg/m^2^, n (%)	3 (3)	27 (19)	< 0.05
Systolic blood pressure, mmHg	122 ± 14	129 ± 20	< 0.05
Diastolic blood pressure, mmHg	72 ± 11	74 ± 12	0.27
Heart rate, bpm	67 ± 11	75 ± 12	< 0.05
Echocardiography			
LV end systolic volume, mL	26 ± 9	26 ± 10	0.82
LV end diastolic volume, mL	74 ± 22	75 ± 21	0.68
LV ejection fraction, %	66 ± 5	66 ± 5	0.93
Stroke volume, mL	67 ± 14	63 ± 13	< 0.05
Left atrial volume index, mL/m^2^	26 ± 9	30 ± 9	< 0.05
LV mass index, g/m^2^	71 ± 19	79 ± 21	< 0.05
E/e′	8.4 ± 2.5	10.7 ± 4.0	< 0.05
e′	9.0 ± 3.1	6.0 ± 1.6	< 0.01
Global longitudinal strain, %	20.3 ± 2.0	18.0 ± 2.6	< 0.05

Values are mean ± SD for normally distributed data and median and interquartile range for non-normally distributed data, or n (%)

*DM* diabetes mellitus, *LV* left ventricular, *E* peak early diastolic mitral flow velocity, *e*′ spectral pulsed-wave Doppler-derived early diastolic velocity from the septal mitral annulus

**Table 2:** Baseline characteristics of T2DM patients with and without overweight

	T2DM patients with overweight (n = 70)	T2DM patients without overweight (n = 75)	p value
Clinical data			
Age, years	59 ± 14	61 ± 13	0.31
Female, n (%)	36 (51)	31 (41)	0.22
Body mass index, kg/m^2^	30 ± 4	22 ± 2	< 0.05
Heart rate, bpm	72 ± 13	70 ± 11	0.25
DM duration, years	12 ± 8	10 ± 10	0.31
Hypertension, n (%)	46 (66)	39 (53)	0.11
Dyslipidemia, n (%)	55 (79)	35 (47)	< 0.05
Blood exam and urinary test			
HbA1c, %	8.5 ± 1.6	8.7 ± 2.5	0.53
Low-density lipoprotein, mg/dL	107 ± 31	110 ± 37	0.52
Triglyceride, mg/dl	165 ± 75	138 ± 89	< 0.05
eGFR, mL/min/1.73 m^2^	72 ± 24	77 ± 26	0.24
Medical treatment			
CCB, n (%)	33 (47)	15 (20)	< 0.05
ACEI/ARB, n (%)	41 (59)	30 (41)	< 0.05
β-Blocker, n (%)	7 (10)	6 (8)	0.78
Statin, n (%)	44 (63)	25 (34)	< 0.05
Insulin, n (%)	41 (59)	32 (43)	0.07
DPP-4I, n (%)	38 (54)	39 (53)	0.85
GLP-1RA, n (%)	12 (17)	2 (2)	< 0.05
Sulfonylurea, n (%)	18 (26)	18 (24)	0.84
α-GI, n (%)	12 (17)	17 (23)	0.36
Thiazolidine, n (%)	10 (14)	4 (5)	0.09
Metformin, n (%)	44 (63)	35 (47)	0.06
Echocardiography			
LV end systolic volume, mL	28 ± 10	25 ± 10	0.08
LV end diastolic volume, mL	78 ± 21	72 ± 21	0.13
LV ejection fraction, %	65 ± 5	66 ± 4	0.06
Stroke volume, mL	64 ± 14	62 ± 11	0.34
Left atrial volume index, mL/m^2^	31 ± 9	29 ± 8	0.08
LV mass index, g/m^2^	84 ± 19	75 ± 21	< 0.05
E/e′	11.1 ± 4.0	10.3 ± 4.1	0.26
e′	5.8 ± 1.4	6.3 ± 1.8	0.06
Global longitudinal strain, %	17.0 ± 2.4	18.9 ± 2.6	< 0.05

Values are mean ± SD for normally distributed data and median and interquartile range for non-normally distributed data, or n (%)

*GFR* estimated glomerular filtration rate, *CCB* calcium channel blocker, *ACEI* angiotensin-converting enzyme inhibitor, *ARB* angiotensin II receptor blocker, *DPP-4I* dipeptidyl peptidase-4 inhibitor, *GLP-1RA* glucagon like peptide-1receptor agonist, *α-GI* α-glucosidase inhibitor. Other abbreviations as in Table 1

### Effect of overweight on LV longitudinal myocardial systolic function in T2DM patients

LV longitudinal myocardial systolic function as assessed in terms of GLS was similar for controls with and without overweight (19.8 ± 1.3% vs. 20.4 ± 2.1%, p = 0.34), whereas GLS for T2DM patients with overweight was significantly lower than that for those without overweight (17.9 ± 2.4% vs. 18.9 ± 2.6%, p < 0.05) (Fig. 2).

**Fig. 2:** Bar graphs showing comparison between global longitudinal strain (GLS) of subjects with and without overweight, showing that GLS of overweight diabetes mellitus (DM) patients is significantly lower than that of non-overweight DM patients, whereas GLS was similar for normal controls with and without overweight

### Association of GLS with overweight in T2DM patients

GLS significantly correlated with BMI in the case of T2DM patients, but no such significant correlation was observed in controls (Fig. 3). Table 3 shows the results of the multiple regression analysis for the association of GLS with clinical and echocardiographic parameters for T2DM patients. An important finding of the multiple regression analysis was that BMI in the case of T2DM patients was the independent determinant parameters for GLS as well as LV volume index.

**Fig. 3:** Dot plots of the association of global longitudinal strain (GLS) with body mass index (BMI), showing significant correlation of GLS with BMI in diabetes mellitus (DM) patients, but no such significant correlation in normal controls

**Table 3:** Multiple regression analysis for GLS in T2DM patients

	Standardizing coefficient	t value	p value
Age	0.019	1.169	0.245
Female	0.144	0.386	0.700
Hypertension	0.295	0.705	0.482
Dyslipidemia	0.481	1.184	0.238
HbA1c	− 0.124	− 1.458	0.157
Body mass index	− 0.147	− 3.600	< 0.001
LV mass index	− 0.053	− 5.193	< 0.001
LA volume index	− 0.015	− 0.585	0.559

R^2^-adjusted: 0.315

F ratio: 9.215 p < 0.001

Abbreviation as in Tables 1 and 2

## Discussion

The findings of the present study indicate that LV longitudinal myocardial systolic function in T2DM patients with overweight was significantly worse than that in T2DM patients without overweight, whereas, no such finding was obtained for age-, gender-, and LVEF-matched controls. In addition, BMI was the independent determinant parameters for GLS for T2DM patients.

### Association of DM-related cardiac dysfunction with HFpEF

HFpEF, which clinically presents as LV diastolic dysfunction, currently accounts for roughly half of all HF cases and its prevalence relative to HFrEF continues to rise at an alarming rate of 1% per year [25]. Patients with HFpEF has similar risk of rate of rehospitalization and mortality as those with HFrEF, which was 5–20 and 3–9% at 30 days, respectively [26, 27]. Patients with HFpEF usually are of advanced age and predominantly women with multiple comorbidities such as hypertension, DM, overweight/obesity, coronary artery disease, atrial fibrillation, hyperlipidemia, renal insufficiency, and sleep apnea [2, 3]. Of these comorbidities, DM is considered a major cause of HFpEF with a prevalence of 20–45% [4]. Thus, DM-related cardiac dysfunction is currently defined as a form of LV diastolic dysfunction, and several studies of DM patients have identified LV diastolic dysfunction as the earliest functional alteration in the course of diabetic cardiomyopathy [5–7], resulting in its establishment as an important prognostic parameter [6]. In fact, LV diastolic dysfunction has been reported as present in 23 to 75% of patients with DM [6, 28, 29].

LV longitudinal myocardial systolic dysfunction, on the other hand, as assessed in terms of lower GLS, has been identified in DM patients with preserved LVEF and without overt coronary artery disease or HF [9–16]. Nakai et al. [10] reported that GLS in DM patients was significantly lower than that in age-matched normal subjects in spite of similar LVEF, and 43% of DM patients showed LV longitudinal myocardial systolic dysfunction detected as GLS < 17.2%. In addition, Ernande et al. [12] showed that 23% of T2DM patients with preserved LVEF had LV longitudinal myocardial systolic dysfunction detected as GLS < 18%. Our group recently demonstrated that, in contrast to age-related LV diastolic dysfunction in normal subjects, LV diastolic function was associated with LV longitudinal myocardial systolic function independently of age in asymptomatic DM patients with preserved LVEF and without coronary artery disease [24]. In addition, recent investigators have maintained that LV longitudinal myocardial systolic dysfunction, rather than LV diastolic dysfunction, may be considered as the first marker of a preclinical form of DM-related cardiac dysfunction in DM patients with preserved LVEF and without overt HF [9, 17]. Ernande et al. further showed that LV longitudinal myocardial systolic dysfunction detected as GLS < 18% was present even in T2DM patients with preserved LVEF and normal LV diastolic function [9]. In addition, our group recently showed that GLS was a strong determinative factor for e′ and E/e′ independent of age or other clinical factors in 177 asymptomatic DM patients with preserved LVEF [24].

### Overweight/obesity and LV diastolic function and HFpEF

Multiple studies have established overweight/obesity as a risk factor for the development of HF. Moreover, recent studies have shown that 29–40% of patients with HF are overweight and 30–49% are obese, with a significantly higher prevalence of obesity for patients with HFpEF compared with patients with HFrEF [30, 31]. It has been also demonstrated that overweight/obesity is an important cause of HFpEF as well as of DM, with more than 80% of patients with HFpEF being overweight/obese [18]. Ichikawa et al. [32] reported their findings from 148 asymptomatic patients with T2DM with preserved LVEF that abdominal visceral adipose tissue as measured by computed tomography was associated with, as well as an independent determinant of, LV diastolic function. Ho et al. [33] also showed that greater BMI was associated with worse GLS in 6231 participants. They also showed that higher circulating leptin concentrations were associated with worse GLS, suggesting a potential role for circulating adipokines in obesity-related LV damage. Although the relationship between overweight/obesity and incident HF may be associated with hemodynamic and anatomic cardiac changes related to excess body mass, recent evidence suggests that the relationship is also mediated by obesity-related inflammatory response, metabolic and insulin resistance, and hormonal changes. Increased inflammatory cytokines such as interleukin-6, interleukin-8 and monocyte chemoattractant protein-1 have been shown to be significant indicators of a greater degree of HFpEF [34]. In addition, high plasma levels of tumor necrosis factor-α and interleukin-6 might cause cardiac diastolic dysfunction by reducing diastolic calcium reuptake in myocytes [35].

Several investigators have reported the association of weight loss with LV diastolic function in obese patients. Karimian et al. [36] reported that weight loss was associated with a reduction in mitral inflow A-wave velocity (from 65.8 ± 19.2 cm/s to 57.0 ± 16.8 cm/s), and an increase in E/A ratio (from 1.2 ± 0.4 to 1.4 ± 0.5) in 32 obese patients (BMI: 40.3 ± 6.6 kg/m^2^) who underwent a 12-week low-calorie fasting phase of a formula die. Furthermore, in eight obese patients with T2DM (BMI: 44 ± 9 kg/m^2^) who underwent sleeve gastrectomy, GLS improved from 13.2  ±  3.7% to 19.7  ±  2.2% (p  <  0.001) and E/e′ also improved from 12 ± 4 to 9 ± 3 (p = 0.028) after surgery [37].

### Effect of overweight/obesity on LV structure

De Jong et al. [38] used 353 patients which were grouped based on diagnosis of obesity, T2DM and hypertension, with normotensive obese patients further separated based on metabolic health. They showed that metabolically healthy normotensive obese patients exhibited relatively low risk of LV concentric remodeling and concentric hypertrophy, whereas, normotensive metabolically non-healthy obese, T2DM and obese/T2DM patients were associated with increased LV concentric remodeling. Furthermore, normotensive patients with both obesity and T2DM had a higher incidence of LV concentric hypertrophy and grade III LV diastolic dysfunction than normotensive patients with either condition alone. Markus et al. [39] also showed that an increase in fat mass was associated with LV concentric remodeling as well as impairment of LV diastolic functional parameters such as E/A ratio and isovolumetric relaxation time in 1189 subjects. Kishi et al. [40] reported that high insulin resistance was associated with worse relative wall thickness and worse peak longitudinal strain and early diastolic strain rate from apical 4-chamber view, and e′, depending on obesity level from 3179 participants. Moreover, Evin et al. [41] showed that left atrial strain as assessed by cardiac magnetic resonance imaging was a sensitive tool for the detection of early LV diastolic dysfunction in individuals with obesity and T2DM and correlated with BMI and epicardial fat. In this study, LV mass index and left atrial volume index in T2DM patients with overweight were significantly larger than those in T2DM patients without overweight (79 ± 21 g/m^2^ vs. 71 ± 19 mg/m^2^, p < 0.05; 30 ± 9 mL/m^2^ vs. 30 ± 9 mL/m^2^, p < 0.05, respectively). On the other hand, LV mass index and left atrial volume index in controls were not different between with overweight and without overweight. (69 ± 14 g/m^2^ vs. 71 ± 19 mg/m^2^, p = 0.62; 25 ± 7 mL/m^2^ vs. 27 ± 9 mL/m^2^, p = 0.39). These differences were thought to be due to the presence of LV subclinical dysfunction as assessed by lower GLS.

### Potential clinical implication of weight loss for T2DM patients

Unlike findings for HFrEF, large trials testing neurohumoral inhibition have consistently failed to attain positive primary outcomes for patients with HFpEF by using, among others, angiotensin-converting enzyme inhibitors, angiotensin II receptor blockers, β-blockers and mineralocorticoid receptor antagonists, thus leading to a poor prognosis for patients with HFpEF [42]. In our study, LV diastolic function as assessed by E/e′ was similar for T2DM patients, both with and without overweight (11.1 ± 4.0 vs. 10.3 ± 4.1, p = 0.26), as well as for controls with and without overweight (8.8 ± 2.8 vs. 8.1 ± 2.8, p = 0.28). These findings were thought to be due to our study population consisting of T2DM patients with asymptomatic status and without a previous history of HF. On the other hand, we were able to show that the association of overweight with LV longitudinal myocardial systolic function was stronger for T2DM patients than for non-DM patients. Moreover, BMI was identified as the independent determinant parameters for LV longitudinal myocardial systolic function in T2DM patients. As explained earlier, LV longitudinal myocardial systolic dysfunction, rather than LV diastolic dysfunction, may be considered the first marker of a preclinical form of DM-related cardiac dysfunction, and the coexistence of LV longitudinal myocardial systolic dysfunction with LV diastolic dysfunction may lead to HFpEF in asymptomatic T2DM patients with preserved LVEF. Obesity/overweight are associated with LV dysfunction and increased risk of HF and other cardiovascular diseases in even general population. However, asymptomatic patients with T2DM and preserved LVEF had impaired GLS compared to age-, gender-, and LVEF-matched non-T2DM subjects, suggesting that patients with T2DM can be particularly susceptible to harm from obesity/overweight. Our findings therefore indicate that the strict control of overweight could be associated with not only improvement of glycemic control, but also prevention of future development of HFpEF in T2DM patients, although the difference of GLS was small in this study.

### Study limitations

This study was a single-center cross-sectional study, so that further longitudinal-based cohort studies are required to validate our results. Another limitation is that no long-term clinical outcome data was not available for this study. For a follow-up of this study, however, long-term clinical data is now being collected for validation of our findings through long-term follow-up studies of the associations of T2DM and overweight with the development of HFpEF in patients with T2DM patients. In addition, the blood examination in a control group such as plasma glucose or lipid data were not part of this study. Finally, the prevalence and degree of obesity in our study was mild compared to that in previous studies from Western countries. This is accounted for by the fact that many obese Asian subjects, including Japanese, show a lesser degree of adiposity than that observed in Western countries [43, 44]. However, Japanese subjects with even mild obesity tend to have obesity-related complications, and The Japanese Committee reported that the relative risk of negative health consequences of obesity in the groups with a BMI of 25.0–26.4 and 26.5–29.9 kg/m^2^ was calculated as 2.5- and 3.9-fold, respectively, of the risk of those with a BMI < 25 kg/m^2^ [45].

## Conclusions

Overweight has a greater effect on LV longitudinal myocardial systolic function in T2DM patients than on that in non-DM healthy subjects. Our finding further suggests that the strict control of overweight in T2DM patients may be associated with prevention of the development of HFpEF.

## Abbreviations

A: late diastolic atrial wave velocity
BMI: body mass index
DM: diabetes mellitus
E: early diastolic trans-mitral flow wave velocity
e′: spectral pulsed-wave Doppler-derived early diastolic velocity from the septal mitral annulus
GLS: global longitudinal strain
HF: heart failure
HFpEF: heart failure with preserved ejection fraction
HFpEF: heart failure with reduced ejection fraction
LV: left ventricular
LVEF: left ventricular ejection fraction
